# The Effect of Humanistic Care Combined with Predictive Nursing on Negative Emotions and Incidence of Cardiovascular Events in Hemodialysis Patients

This article has been retracted.

**DOI:** 10.1155/2022/7562525

**Published:** 2022-04-29

**Authors:** Yanling Wang, Changmin Su

**Affiliations:** Department of Blood Purification Center, The First People's Hospital of Lianyungang, Lianyungang, Jiangsu 222000, China

## Abstract

**Objective:**

To explore the effect of humanistic care combined with predictive nursing on the negative emotions and incidence of cardiovascular events in hemodialysis patients.

**Methods:**

A total of 90 patients undergoing hemodialysis in our hospital from December 2020 to September 2021 were selected as the research subjects and divided into the study group (*n* = 45) and the control group (*n* = 45) by the random number table method. The patients in the control group were given routine nursing, and the patients in the study group were given humanistic care combined with predictive nursing. The effects between the two groups were compared.

**Results:**

After nursing, cardiac troponin I (cTn I) level, Hamilton Depression Scale (HAMD) scores, and Hamilton Anxiety Scale (HAMA) scores in the two groups decreased, and the scores were lower in the study group than the control group (*P* < 0.05). The World Health Organization on Quality of Life Brief Scale (WHOQOL-BREF) scores in both groups increased and were higher in the study group than the control group (*P* < 0.05). The nursing satisfaction in the study group was higher than that in the control group, and the incidence of cardiovascular adverse events in the study group was lower than that in the control group (*P* < 0.05).

**Conclusion:**

In the process of hemodialysis, the application of humanistic care combined with predictive nursing to hemodialysis patients can significantly decrease the cTn I level, reduce the negative emotions of patients, improve the quality of life and nursing satisfaction of patients, and reduce the occurrence of adverse cardiovascular events.

## 1. Introduction

At present, the most commonly used clinical treatment method of end-stage renal disease is hemodialysis, which can effectively improve the quality of life of patients, prolong the life cycle, and has important clinical significance in improving the prognosis of patients [1, 2]. However, during the clinical treatment of hemodialysis, glucose can be lost, and the decline in renal function will in turn act on exogenous insulin, causing its degradation rate to slow down, causing the ineffectiveness of hemodialysis treatment in removing macromolecular substances. Thus, patients are prone to hypoglycemia and even have adverse events such as cardiovascular and cerebrovascular diseases, which seriously threaten the life safety of patients [3]. Professional nursing can reduce complications, prolong service time, and improve life quality for renal failure patients during hemodialysis [4]. Therefore, it is very important to enhance the nursing quality for hemodialysis patients, pay attention to the changes of their physical conditions, and be alert to the occurrence of complications. Although routine nursing can alleviate the clinical symptoms of patients, its effect is not ideal. Humanistic care is to put the concept of “patient-centered” service into clinical application, so as to truly serve patients. However, with the prolongation of hemodialysis, the incidence of complications also tends to increase, which not only affects the dialysis process but also causes the unfavorable prognosis of patients. Therefore, this study adopted humanistic care combined with predictive nursing. The negative emotions and incidence of cardiovascular events in hemodialysis patients were observed.

## 2. Materials and Methods

### 2.1. General Data

A total of 90 patients undergoing hemodialysis in our hospital from December 2020 to September 2021 were selected as the research subjects and divided into the study group (*n* = 45) and the control group (*n* = 45) by the random number table method. The study was approved by the medical ethical committee of the First People's Hospital of Lianyungang. Inclusion criteria were the following: (1) those who were diagnosed with end-stage renal disease by clinical or laboratory tests [5], (2) those who had clear mind and could coordinate the treatment, (3) those who were expected to live for more than half a year, (4) those who were physically able to tolerate hemodialysis, (5) those who were not complicated by severe hepatobiliary diseases, and (6) those who had complete clinical data. Exclusion criteria were the following: (1) those with autoimmune diseases or coagulation disorders, (2) those with a history of cardiovascular disease, (3) those with malignant tumors, (4) those with infection or susceptibility before enrollment, and (5) pregnant or lactating women.

### 2.2. Methods

The patients in the control group were given routine nursing. The patients in the study group were given humanistic care combined with predictive nursing.

*Humanistic care*: (1) environmental nursing: for newly admitted patients, nursing staff took the patients for a walk in the hospital in free time to make them get familiar with the hospital environment as soon as possible. Patients were provided with a warm and comfortable ward during hospitalization to eliminate fear and feel cared. For patients with hyperkalemia, nurses were supposed to strengthen ward rounds to detect various abnormal conditions in time to avoid serious consequences. If patients were accompanied by hyperkalemia, nurses were supposed to greet as many times as possible to avoid serious consequences. (2) Psychological nursing: because hemodialysis treatment is a long process, patients might be troubled by emotions such as fear, and nurses were supposed to communicate with patients as much as possible and timely find out the problems encountered by patients during treatment or other periods and make a prompt response. (3) Life nursing: during hemodialysis, nurses were supposed to protect the privacy of patients and respect the ideas of patients, so as to better communicate with patients. Nurses adjusted the temperature and humidity of the ward according to the patients' demands. The night nursing staff were supposed to avoid making excessive noise. (4) Social relationship nursing: due to the long process of hemodialysis treatment, family members might have some negative emotions that affected the patients' optimistic attitudes towards the disease. Nursing staff were supposed to make family members and patients understand the disease by distributing brochures or TV education, etc., and informed family members that the support of family members was of great significance to the patients' condition and mentality. Nursing staff were encouraged to regularly hold social gatherings, birthday parties, etc., for patients to alleviate the patients' negative psychological state. (5) Dietary nursing: during hemodialysis treatment, patients needed to maintain a light diet. Nursing staff could work with the health manager of the hospital to formulate detailed recipes for patients, pay attention to low-protein diets, prohibit smoking and drinking, etc.

*Predictive nursing*: a nursing team of 6 to 8 nursing staff was led by an experienced head nurse, and then, a one-week skill training was conducted. After passing the assessment, they could participate in the study. Nurses predicted possible adverse conditions in the hemodialysis process, such as hypotension, angina pectoris, myocardial infarction, and heart failure, by consulting relevant information, previous nursing experience, etc., and preset one or more prevention and treatment measures for various adverse conditions.

### 2.3. Observation Indicators

(1) General data include gender, age, body mass index (BMI), disease type, and education level. (2) Cardiac troponin I (cTn I) level: 5 mL of fasting venous blood was drawn in the morning, centrifuged at 3000 r/min for 10 min, and the supernatant was taken. The cTn I level was detected by the automatic chemiluminescence method using an ACCESS 2 Immunoassay System analyzer (Beckman Coulter, USA). (3) Negative emotion scoring: the Hamilton Depression Scale (HAMD) [6] and the Hamilton Anxiety Scale (HAMA) [7] were used for evaluation. The HAMD contained a total of 17 items: total score below 7: normal; 8 points < total score < 17 points: mild depression; 18 points < total score < 24 points: moderate depression; and total score ≥ 25 points: severe depression. The HAMA consisted of 15 items, with a total score of 45 points. The higher the score, the more anxious the patients. (4) Quality of life scoring: the World Health Organization on Quality of Life Brief Scale (WHOQOL-BREF) [8] was used to evaluate the quality of life of patients. The scale included 4 items of social relationship, physiological domain, social environment, and psychological domain, with a total score of 26 to 130 points. The higher the score, the better the quality of life of the patients. (5) Nursing satisfaction: at the end of hemodialysis treatment, a hospital-made satisfaction questionnaire was face to face issued to patients or their families to evaluate the service of nursing staff, including service attitude, professional knowledge and skills, and ability to handle critical events. The results could be satisfied, basically satisfied, and dissatisfied. The patients or their families filled in the questionnaire in the absence of the nursing staff and returned the questionnaire into a questionnaire bin. (6) Adverse cardiovascular events including arrhythmia, angina pectoris, myocardial infarction, heart failure, and cardiac death during hospitalization were evaluated.

### 2.4. Statistical Analysis

SPSS 24.0 software was used to analyze and process the data of this study. The measurement data was expressed as *x* ± *s*, and the *t* test was used. The count data was expressed as %, and the *χ*^2^ test was used. *P* < 0.05 indicated that the difference was statistically significant.

## 3. Results

### 3.1. Comparison of General Data between the Two Groups

There were no significant differences in general data between the two groups (*P* > 0.05), as shown in Table 1.

### 3.2. Comparison of cTn I Level between the Two Groups

After nursing, the cTn I level in both groups decreased. The cTn I level was lower in the study group than the control group (*P* < 0.05), as shown in Table 2.

### 3.3. Comparison of Negative Emotion Scores between the Two Groups

After nursing, the negative emotion scores in both groups decreased (*P* < 0.05). HAMD and HAMA scores were lower in the study group than the control group (*P* < 0.001), as shown in Table 3.

### 3.4. Comparison of Quality of Life Scores between the Two Groups

After nursing, the WHOQOL-BREF scores in both groups increased, and the study group was higher than the control group (*P* < 0.05), as shown in Table 4.

### 3.5. Comparison of Nursing Satisfaction between the Two Groups

The nursing satisfaction in the study group was significantly higher than that in the control group (*P* < 0.05), as shown in Table 5.

### 3.6. Comparison of Adverse Cardiovascular Events between the Two Groups

There were 4 cases of angina pectoris, 2 cases of arrhythmia, and 1 case of chronic heart failure in the control group, with an incidence of 15.56%. There was only 1 case of arrhythmia in the study group, which was cured after treatment, with an incidence of 2.2%, which was significantly lower than that in the control group (*P* < 0.05), as shown in Table 6.

## 4. Discussion

In recent years, with the rapid development of social life, people's lifestyles and habits have also undergone significant changes, which has also led to increase in the incidence of end-stage renal disease, posing a serious threat to the life safety of patients [9]. Therefore, active treatment is essential for improving the quality of life of patients.

Hemodialysis is to purify the blood through the filtration of semipermeable membranes, thereby maintaining the acid-base and electrolyte balance in the body and protecting the residual renal function of patients [10]. However, due to the long process of this treatment and the need to limit the patients' position during the treatment process, the blood drainage out of the body for circulation is blocked, resulting in a sharp decrease in the blood volume of the body. Therefore, cardiovascular events are easily caused during the treatment period, which affects the treatment process and prognosis of the patients [11]. Therefore, giving special nursing in the course of treatment has far-reaching significance in changing the prognosis of patients.

Under the influence of the value of serving the people, the hospital has paid more and more attention to the construction of spiritual civilization. Humanistic care is a “people-oriented, patient-centered” nursing model that improves patients' life, psychological state, and emotion on the basis of routine nursing. It makes patients willing to cooperate with the treatment and alleviate the tension between doctors and patients to some extent, thereby improving the quality of nursing. Predictive nursing, also known as advanced nursing or prenursing, is an emerging nursing model that requires nurses to conduct a comprehensive assessment of the patients' condition in advance, predicts possible complications in the treatment process based on past experience, and then strengthens nursing procedures to improve the prognosis of the patients. This nursing mode can make nursing staff change from routine passive nursing to active nursing, which can not only improve the ability of nursing staff to predict and infer but also ensure patients' safety to a certain extent, targeted, purposeful, and comprehensive.

Long-term hemodialysis can cause a variety of complications and adverse events while treating diseases, among which cardiovascular disease is the most common [12]. cTn I is a contractile protein that exists only in cardiomyocytes and has high specificity. When cardiomyocytes are damaged or necrotic, cTn I is released into the blood due to its small molecular weight and enters the blood circulation of the body to increase its content in serum and thus is currently the best sensitive marker of myocardial injury in clinical practice [13]. The results of this study showed that the cTn I level in the study group was significantly lower than that in the control group, and the incidence of cardiovascular adverse events was lower than that in the control group, indicating that the application of humanistic care combined with predictive nursing during hemodialysis treatment can reduce the serum cTn I level of patients and then reduce the incidence of cardiovascular adverse events, similar to the results of a previous study [14]. The reasons may be related to the early prediction and treatment of adverse events during hemodialysis by predictive nursing through relevant clinical experience, patients' condition, medical records, etc., so as to improve the cTn I level in patients and reduce the occurrence of cardiovascular events to a certain extent [15].

The results of this study showed that there were no significant differences in the scores of HAMA and HAMD between the two groups before nursing; after nursing, the scores of HAMA and HAMD in the two groups decreased and those in the study group were lower; the scores of WHOQOL-BREF in both groups increased after nursing and were higher in the study group than the control group [16, 17], indicating that both nursing modes can eliminate or improve the negative emotions of patients, while humanistic care combined with predictive nursing can minimize the negative emotions of patients, improve patients' treatment compliance, and then improve the quality of life of patients. In addition, the patients in the study group were significantly more satisfied with nursing than those in the control group. It may be related to the fact that humanistic care combined with predictive nursing can predict complications and to a certain extent enhance the patients' or family members' awareness of the disease, and strengthening communication between doctors and nurses can bring doctors and patients closer. Through encouragement, etc., it can help patients to improve their confidence in the recovery or improvement of the disease, maintain a positive and optimistic attitude, and thus improve the nursing satisfaction of patients or their family members.

## 5. Conclusion

The application of humanistic care combined with predictive nursing can reduce the serum cTn I level of patients to a certain extent during hemodialysis, thereby decreasing the occurrence of cardiovascular adverse events; reducing negative emotions such as anxiety, depression, etc.; and improving the quality of life and nursing satisfaction.

## Figures and Tables

**Table 1:** General data in the two groups.

General data	Control group (*n* = 45)	Study group (*n* = 45)	*χ* ^2^/*t*	*P*
Gender (*n* (%))				
Male	23 (51.11)	21 (46.67)	0.178	0.673
Female	22 (48.89)	24 (53.33)		
Age (*x* ± *s*, year)	64.28 ± 5.34	64.51 ± 5.32	0.205	0.838
BMI (*x* ± *s*, kg/m^2^)	23.01 ± 2.17	22.87 ± 2.25	0.300	0.765
Disease type (*n* (%))				
Hypertensive nephropathy	16 (35.56)	17 (37.78)		
Diabetic nephropathy	21 (46.67)	19 (42.22)	0.189	0.910
Glomerulonephritis	8 (17.77)	9 (20.00)		
Educational level (*n* (%))				
Elementary or junior high school	24 (53.33)	19 (42.22)		
Senior high school	18 (40.00)	21 (46.67)	1.312	0.519
College and above	3 (6.67)	5 (11.11)		

**Table 2:** cTn I level in the two groups (*x* ± *s*, ng/L).

Groups	Before nursing	After nursing
Control group (*n* = 45)	53.27 ± 6.21	39.57 ± 3.44^a^
Study group (*n* = 45)	53.36 ± 6.18	31.54 ± 3.15^a^
*t*	0.069	11.549
*P*	0.945	<0.001

Note: versus before nursing, ^a^*P* < 0.05.

**Table 3:** Negative emotion scores in the two groups (*x* ± *s*).

Groups	HAMD scores		HAMA scores	
	Before nursing	After nursing	Before nursing	After nursing
Control group (*n* = 45)	21.08 ± 1.76	15.34 ± 1.23^a^	37.58 ± 4.12	21.45 ± 3.51^a^
Study group (*n* = 45)	21.23 ± 1.85	9.51 ± 1.36^a^	37.88 ± 4.20	14.56 ± 3.21^a^
*t*	0.394	21.328	0.342	9.717
*P*	0.694	≤ 0.001	0.733	≤0.001

Note: versus before nursing, ^a^*P* < 0.05.

**Table 4:** Quality of life scores in the two groups (*x* ± *s*).

Groups	Time	Social relationship	Physiological domain	Social environment	Psychological domain
Control group (*n* = 45)	Before nursing	31.25 ± 2.18	34.17 ± 3.09	38.54 ± 2.86	29.74 ± 2.35
	After nursing	98.43 ± 9.57^a^	93.62 ± 9.49^a^	105.24 ± 9.65^a^	103.41 ± 10.25^a^
Study group (*n* = 45)	Before nursing	30.78 ± 2.31	33.91 ± 3.14	37.89 ± 2.93	29.46 ± 2.54
	After nursing	105.25 ± 9.89^ab^	98.27 ± 9.68^ab^	112.08 ± 10.06^ab^	113.54 ± 10.35^ab^

Note: versus before nursing, ^a^*P* < 0.05; versus the control group, ^b^*P* < 0.05.

**Table 5:** Nursing satisfaction in the two groups.

Groups	Satisfied (*n* (%))	Basically satisfied (*n* (%))	Dissatisfied (*n* (%))	Satisfaction rate
Control group (*n* = 45)	18 (40.00)	15 (33.33)	12 (26.67)	73.33% (33/45)
Study group (*n* = 45)	25 (60.00)	18 (66.67)	2 (4.44)	95.56% (43/45)
*χ* ^2^				8.459
*P*				0.004

**Table 6:** Adverse cardiovascular events in the two groups (*n* (%)).

Groups	Angina pectoris	Arrhythmia	Chronic heart failure	Total
Control group (*n* = 45)	4 (8.89)	2 (4.44)	1 (2.22)	7 (15.56)
Study group (*n* = 45)	0 (0.00)	1 (2.22)	0 (0.00)	1 (2.22)
*χ* ^2^				4.45
*P*				≤0.001

## Data Availability

The data in the current study are available from the corresponding author on reasonable request.
